The article "The Predictive Effect of Negative Psychological Emotions of Anxiety and Depression on the Poor Prognosis of CHD Patients with Stent Implantation and the Improvement of Clinical Intervention Measures" was retracted in 2023. Reasons: signs of a paper mill; compromised peer review; unreliable results or conclusions.

# The Predictive Effect of Negative Psychological Emotions of Anxiety and Depression on the Poor Prognosis of CHD Patients with Stent Implantation and the Improvement of Clinical Intervention Measures

**DOI:** 10.1155/2022/2534277

**Published:** 2022-01-30

**Authors:** Guoxing Li, Yuhuan Tian, Qiumin Zhang, Zhaofeng Jin, Yuping Song

**Affiliations:** Weifang Medical University, Weifang, Shandong 261053, China

## Abstract

**Objective:**

To explore the predictive effect of negative emotions such as anxiety and depression on the poor prognosis of coronary heart disease (CHD) patients with stent implantation and to seek the improvement of clinical intervention measures.

**Methods:**

A total of 303 patients with CHD and PCI were recruited from February 2019 to April 2021. The risk factors of CHD such as anxiety and depression, age, sex, smoking and drinking, BMI, hypertension, diabetes, dyslipidemia, and family history of CHD were collected. Meanwhile, clinical data such as laboratory examination, angiography, diseased vessels, and stent types were collected. The patients were followed up for 1 year, and the medical records, hospitalization records, or death records were checked by telephone interview once a month. Major adverse cardiovascular events (MACE) such as emergency and causes, readmission times and causes, new nonfatal myocardial infarction, stent restenosis, heart failure, arrhythmia, and death were recorded. The incidence of anxiety and depression in patients after PCI was counted, and Cox regression was applied to analyze the influence and prediction of anxiety and depression on MACE in patients with CHD stent implantation and improve clinical intervention measures.

**Results:**

Compared with those without MACE, anxiety (56.25% vs 30.63%), depression (62.5% vs 22.88%, *P* < 0.01), anxiety combined with depression (46.88% vs 15.50%, *P* < 0.01), and hypertension history (71.8% vs 39.11%, *P* < 0.01) were more common in patients with MACE. Uncorrected Cox proportional hazard regression found that people with anxiety had a higher risk of developing MACE than those without anxiety (HR 3.181, *P* < 0.01). Multiple Cox proportional hazard regression analysis of anxiety showed that anxiety was an independent predictor of cumulative MACE (*P* < 0.01). The risk of developing MACE in patients with anxiety was 3.742 times higher than that in patients without anxiety (*P* < 0.01). Uncorrected Cox hazard regression analysis showed that people with depression had a higher risk of developing MACE than those without depression (HR 5.434, *P* < 0.01). Furthermore, the results also uncovered that depression was an independent predictor of cumulative MACE (*P* < 0.01). The risk of MACE in patients with depression was 3.087 times higher than that in patients without depression (*P* < 0.01). Cox hazard regression showed that the risk of MACE in patients with anxiety and depression was significantly higher than that in patients without anxiety and depression (HR 4.642, *P* < 0.01). After screening, it was found that anxiety with depression could predict the occurrence of MACE (*P* < 0.01). The risk of MACE in patients with anxiety and depression was 3.702 times higher than that in patients without anxiety and depression (*P* < 0.01). Cox regression analysis showed that the risk of MACE with only anxiety and depression was 2.793 times higher than that without anxiety and depression (95% CI 0.914 8.526), with no statistical significance (*P* > 0.05), and the risk of MACE with depression without anxiety was significantly higher than that without anxiety and depression (*P* < 0.01). The risk of MACE in patients with anxiety and depression was 7.303 times higher than that in patients without anxiety and depression (*P* < 0.01).

**Conclusion:**

Negative emotions such as anxiety and depression can increase the risk of poor prognosis of patients with CHD. Therefore, in clinical work, in addition to routine treatment and nursing during hospitalization, it is recommended to screen patients with depression in CHD patients. Medical staff should use simple and effective assessment tools in time and take active measures to improve the depression of patients. This trial is registered with ChiCTR2200055645.

## 1. Introduction

Coronary heart disease (CHD) is a major disease that threatens human life and health, which is also one of the leading causes of death of patients [1–3]. The prevalence rate of CHD in China is increasing year by year, and the case fatality rate continues to increase, resulting in the aggravation of social and economic burden and the serious decline of people's health quality. Prevention and treatment of CHD, reduce its incidence and mortality, improve prognosis, has become one of the central topics in the global cardiovascular field. Percutaneous coronary intervention (PCI) is widely used in the treatment of CHD. Over the past few years, although improvements in some therapeutics, such as drug-eluting stent usage, have reduced coronary artery restenosis and thrombosis from 30%–40% to 15% one year after PCI, restenosis and thrombosis are still serious clinical problems [4–7]. Therefore, it is still necessary to actively control the risk factors of CHD in order to prevent the occurrence of major adverse cardiovascular events (MACEs). So far, age, sex, hypertension, dyslipidemia, diabetes, smoking, obesity, family history, degree of vascular stenosis, and C-reactive protein (CRP) levels have been confirmed to be risk factors for MACE in patients with CHD but these factors cannot fully explain the development of CHD. In recent years, more and more attention has been paid to the role of psychological factors, especially anxiety and depression, in the occurrence and development of CHD. Heart attack and PCI surgery itself as stressors make patients aware of the threat of their own disease to life, resulting in many patients with anxiety and depression after PCI, while anxiety and depression can reduce patients' compliance with treatment and greatly reduce their clinical benefits [8–10]. Based on this, this study surveyed the value of anxiety and depression assessment in 303 patients with CHD who underwent PCI stent implantation in our hospital from February 2019 to April 2021. The results and conclusions are as follows.

## 2. Patients and Methods

### 2.1. General Information

A total of 303 patients with CHD who underwent PCI stent implantation were selected from February 2019 to April 2021. The clinical data of anxiety and depression, age, sex, smoking and drinking status, BMI, hypertension, diabetes, dyslipidemia, family history of premature CHD, disease diagnosis, laboratory examination, angiography, diseased vessels, stent types, and other risk factors of CHD were collected. The age of all patients ranged from 53 to 74 years, with an average of 66.91 ± 3.63 years. This study was approved by the requirements of our school, and all patients signed informed consent.

Patients were excluded from the study under the following circumstances: (1) surgical treatment; (2) patients who were diagnosed with anxiety and/or depression or other mental disorders or were treated with antianxiety, depressive drugs, or other mental disorders before admission; (3) patients who had previously undergone coronary artery revascularization; and (4) complicated with other severe diseases such as tumor and vital organ failure.

### 2.2. Follow-Up Method

#### 2.2.1. Baseline Data Survey and Indicator Determination

Train all investigators before starting the investigation. During the survey, the purpose and method of the study were explained to the subjects in advance and consent was obtained. Blood samples were collected within 24 hours before PCI for measurement of echocardiography from 1 to 4 days after hsCRP, PCI. Anxiety status and depression status were measured by the hospital anxiety and depression scale. The investigators used unified instructions to investigate, and the questionnaires were distributed and collected on the spot. The demographic and clinical data needed by the subjects were obtained by the researchers asking the subjects and consulting the medical records.

#### 2.2.2. Follow-Up of MACE after Discharge

Within one year after discharge, the patient was followed up by a trained competent nurse by telephone once a month and the occurrence of MACE was obtained. Any adverse events reported by the patient were verified by outpatient and emergency medical records, hospitalization records, examination reports, or death certificates. When my statement is unclear due to older age, low education, or other reasons, check with his main caregiver and consult the medical records. When unable to contact me, contact me through the telephone number or home address of the main contact person left at the time of admission.

### 2.3. Observation Indicators and Projects

#### 2.3.1. General Situation Questionnaire

On the basis of consulting the literature and consulting relevant experts, the research group compiled the questionnaire on the general situation of this study, including the demographic data of patients' age, sex, marital status, education, occupation, and income. Meanwhile, it also included the height, weight, smoking, drinking, hypertension, diabetes, history of dyslipidemia, family history of premature CHD, disease diagnosis, PCI indication (emergency or elective PCI), number of diseased blood vessels, degree of coronary artery stenosis, number of stents, type of stents, and mental health status, including history of mental illness and use of psychotropic drugs.

#### 2.3.2. Hospital Anxiety and Depression Scale (HADS) [11]

HADS was compiled by Zigmond AS and Snaith RP in 1983 and is mainly used for patients in general hospitals [12]. The scale has 14 items, including 2 subscales of anxiety and depression, 7 items for anxiety and 7 for depression. 0–3 is a grade score, that is, the highest score of anxiety and depression is no more than 21 points, and the lowest score is 0 points. The anxiety subscale was 1, 3, 5, 7, 9, 11, and 13, and the depression subscale was 2, 4, 6, 8, 10, 12, and 14. In the anxiety subscale, the 7th item was scored in reverse and the 2nd, 4th, 6th, 12th, and 14th items in the depression subscale were scored in reverse. According to the standard of the original author of the scale, the total score of 0–7 of the two subscales represents no anxiety or depression, the total score of 8–10 represents possible or critical anxiety or depression, and the total score of 11–21 represents obvious anxiety or depression. Take 8 points as the starting point, that is, including those who are suspicious and those with symptoms which are all positive. Cronbach's *α* coefficient of anxiety subscale was 0.92 and Cronbach's *α* coefficient of depression subscale was 0.84.

#### 2.3.3. hsCRP

Venous blood was collected after fasting within 24 hours before PCI, and the level of hsCRP was measured by hypersensitive immunoassay-latex agglutination (N-high sensitivity hsCRP).

#### 2.3.4. MACE Questionnaire

The study group developed a MACE questionnaire to record the number of emergency visits and causes, rehospitalization times, and causes of patients with CAD stent implantation during the follow-up period. Nonfatal new myocardial infarction, in-stent restenosis, repeated revascularization (PCI or CABG), angina pectoris, arrhythmia, heart failure, and death were collected. MACE includes angina pectoris, nonfatal new myocardial infarction, heart failure, arrhythmia, in-stent restenosis, repeated revascularization (PCI or CABG), and death (judged by death certificate issued by the hospital or public security organ). The occurrence of any of the above adverse events is the end point of follow-up. The time from the stent implantation to the occurrence of the first MACE was calculated as the outcome index. Some adverse cardiovascular events are defined as follows: (1) angina pectoris: typical angina pectoris occurs again after PCI, characterized by retrosternal or precordial pain during activity or rest, which usually lasts no more than 20 minutes; ST-T changes are found in ECG during attack, and there is no increase in myocardial injury markers; (2) myocardial infarction: patients with recurrent myocardial injury markers cTnT and/or CK-MB exceeding 99% percentile from 24 hours after PCI to the end of follow-up, evidence of myocardial ischemia and one of the following: ischemic symptoms; elevation of ST segments in two or more adjacent leads of ECG beyond lmm, or new left bundle branch block; new pathological Q wave on ECG. The imaging examination showed that there was a new stage of abnormal wall motion; (3) heart failure: dyspnea occurred after PCI, including exertional dyspnea, orthopnea, nocturnal paroxysmal dyspnea, New York heart function grade ≥ 3, signs of pulmonary edema or peripheral edema, ventricular enlargement, and systolic insufficiency by echocardiography; and (4) arrhythmia refers to severe ventricular arrhythmias (polymorphic ventricular premature, paroxysmal ventricular tachycardia, torsade ventricular tachycardia, ventricular flutter, and ventricular fibrillation) with hemodynamic instability and first atrial flutter, atrial fibrillation, and supraventricular tachycardia.

### 2.4. Statistical Analysis

SPSS23.0 statistical software was used for statistical analysis, and the measurement data were represented by $\bar{x}\pm s$. Normal distribution and homogeneity of variance were tested before statistical analysis. The *t*-test was used to compare the two groups, *n* (%) was used to represent the counting data, and *χ*^2^ test was used to analyze the counting data. The difference was statistically significant (*P* < 0.05).

## 3. Results

### 3.1. Univariate Analysis of the Incidence of MACE in Patients with CHD after Stent Implantation

Compared with patients without MACE, patients with MACE had more anxiety (56.25% vs 30.63%), depression (62.5% vs 22.88%, *P* < 0.01), anxiety with depression (46.88% vs 15.50%, *P* < 0.01), and history of hypertension (71.8% vs 39.11%, *P* < 0.01). All the data are shown in Tables 1 and 2.

### 3.2. Analysis of the Influence of Anxiety on MACE

Through the proportional hazard regression analysis of Cox, it was found that the risk of MACE in anxiety patients was higher than that in nonanxiety patients (HR 3.181, 95% CI 1.603~6.301, *P* < 0.01). Demographic and clinical data including age, sex, BMI, smoking, hypertension, diabetes, dyslipidemia, family history of premature CHD, number of diseased vessels, degree of stenosis of diseased vessels, LVEF, and hsCPR (Table 2 of variable assignment) were included. Multiple Cox proportional hazard regression analysis of anxiety showed that anxiety was an independent predictor of cumulative MACE. The risk of MACE in patients with anxiety was 3.742 times higher than that in patients without anxiety (95% CI 1.518-9.173, *P* = 0.003). All the data are shown in Table 3.

### 3.3. Cox Regression Analysis of the Effect of Anxiety Combined with Depression on MACE

Through Cox proportional hazard regression analysis, it was found that the risk of MACE in patients with anxiety combined with depression was significantly higher than that without anxiety and depression (HR 4.642, 95% CI 2.363~9.104, *P* < 0.01). Age, sex, BMI, smoking, hypertension, diabetes, dyslipidemia, family history of premature CHD, number of diseased vessels, degree of stenosis of diseased vessels, LVEF, and hsCPR were included in multiple Cox proportional hazard regression analysis of anxiety with depression. After screening, it was found that anxiety with depression could predict the occurrence of MACE. The risk of MACE in patients with anxiety and depression was 3.702 times higher than that in patients without anxiety and depression (95% CI 1.576, 8.673, *P* < 0.01). All the data are shown in Table 4.

### 3.4. COX Regression Analysis of the Effect of Anxiety Combined with Depression on MACE

Through Cox regression analysis, it was found that the risk of MACE in patients without anxiety and depression was 2.793 times higher than that in patients without anxiety and depression (95% CI 0.914~8.526) but there was no statistical significance (*P* = 0.075) and the risk of MACE in patients with depression and without anxiety was significantly higher than that in patients without anxiety and depression (HR = 5.734, 95% CI 1.873~17.546, *P* < 0.01). The risk of MACE in patients with anxiety and depression was 7.303 times higher than that in patients without anxiety and depression (95% CI 3.091-17.231, *P* < 0.01). The results are shown in Table 5. From the above results, it can be seen that anxiety alone does not significantly increase the risk of MACE, while depression or anxiety combined with depression increases the risk of MACE.

## 4. Discussion

CHD remains one of the leading causes of death worldwide. In 2008, about 17.3 million people died of cardiovascular disease, accounting for almost 30% of deaths [12–14]. It is estimated that this number will increase to 23.6 million by 2030, mainly in low- and middle-income countries. Meanwhile, the number of patients with psychological disorders is also increasing. According to the World Health Organization (WHO), depression will become the second leading cause of human dysfunction after cardiovascular disease by 2030. About 10% of any age suffer from psychological disorders [15–17]. The high incidence of cardiovascular disease and psychological disorders has provoked an increase in the incidence of psychological disorders in patients with cardiovascular disease. In fact, anxiety and depression are more common in patients with cardiovascular disease than expected. For example, studies have shown that the incidence of depression in patients with CHD is 14%–47%, which is significantly higher than the depression rate of 4%–7% of the total population [18–20]. Even using the Diagnostic and Statistical Manual of Mental Disorders (DSM) with more stringent diagnostic criteria, 20% of patients with CHD can still be detected to have definite depressive symptoms [20].

At present, PCI is one of the main methods for the treatment of CHD. Stent implantation can significantly reduce the somatic symptoms and mortality of patients with CHD. In recent years, the number of patients treated with PCI has increased year by year, forming a large group. However, although PCI treatment can eliminate or relieve the symptoms of CHD, heart attack and PCI surgery themselves act as stressors to make patients aware of the life-threatening threat of CHD. Meanwhile, although the application of drug-eluting stents reduces the incidence of MACE after PCI, stents still have the problems of restenosis and thrombosis. Coupled with the lack of knowledge of the CHD, some patients treated with PCI have anxiety and depression [21, 22]. Some studies have shown that patients treated with PCI are generally accompanied with emotional disorders such as anxiety and depression and the incidence of anxiety and depression is higher than that of patients without PCI treatment [23–25]. A systematic review of the prevalence of depression in patients with CHD in Chinese population shows that the total incidence of depression in patients with CHD is 51%, the incidence of depression in patients living in the community is 34.6% to 45.8%, and that of severe depression is 3.1% to 11.2%. However, the recognition rate of depression in CHD PCI patients is less than 25% [26]. Therefore, there is an urgent need to strengthen the evaluation of the psychological status of patients during hospitalization.

As we know, some patients with CHD have both anxiety and depression. Our present study found that the incidence of anxiety complicated with depression was 18.12%. It has been reported that 18.33% of patients with CHD with severe depression have anxiety at the same time [27–30]. At present, the explanation for the coexistence of anxiety, depression, and CHD is not unified [30]. Some scholars believe that CHD is the basis of the coexistence of both and anxiety and depression are only different manifestations of the CHD [29]. Other scholars believe that anxiety and depression are independent diseases and exist in the population of patients with CHD, while other scholars believe that anxiety and depression is a new type of disease independent of anxiety and depression [30]. This study found that there was more anxiety, depression, anxiety combined with depression, and hypertension history in patients with MACE than those without MACE. Uncorrected Cox proportional hazard regression found that people with anxiety had a higher risk of developing MACE than those without anxiety (HR 3.181~95% CI 1.603~6.301, *P* = 0.001). By multiple Cox analysis of anxiety, it was found that anxiety was an independent predictor of cumulative MACE. The risk of MACE in patients with anxiety was 3.742 times higher than that in patients without anxiety. Uncorrected Cox analysis showed that people with depression had a higher risk of developing MACE than those without depression.

In addition, multiple Cox regression analysis of depression showed that depression was an independent predictor of cumulative MACE in patients (*P* = 0.006). The risk of MACE in patients with depression was 3.087 times higher than that in patients without depression. Cox regression showed that the risk of MACE in patients with anxiety and depression was significantly higher than that in patients without anxiety and depression. Age, sex, BMI, smoking, hypertension, diabetes, dyslipidemia, family history of premature coronary heart disease, number of diseased vessels, degree of stenosis of diseased vessels, LVEF, and hsCPR were included in multiple Cox proportional hazard regression analysis of anxiety with depression. After screening, it was found that anxiety with depression could predict the occurrence of MACE. Patients with anxiety and depression had a 3.702-fold higher risk of developing MACE than those without anxiety and depression. Therefore, anxiety can predict the occurrence of MACE without considering the effects of depression.

However, other studies have revealed that anxiety is not related to the prognosis of CHD. A meta-analysis of 30527 patients included in 44 studies indicated that when other risk factors were not controlled, the risk of death of CHD with anxiety was 1.21 times higher than that with nonanxiety but when other risk factors were controlled, the effect of anxiety on CHD mortality was no longer significant [31]. This study also established the effect of anxiety combined with depression on cardiovascular events in patients with CHD undergoing PCI. The results showed that the risk of MACE with anxiety and depression was 2.793 times higher than that of patients without anxiety and depression but there was no statistical significance (*P* > 0.05). Furthermore, the risk of MACE in patients with depression without anxiety was significantly higher than that without anxiety and depression. The risk of MACE in people with anxiety and depression was 7.303 times higher than that without anxiety and depression (95% CI 3.091-17.231, *P* < 0.001). From the above results, it can be concluded that anxiety alone does not significantly increase the risk of MACE, while depression or anxiety combined with depression increases the risk of MACE, which indicates that depression rather than anxiety is an important predictor of mortality in patients with PCI.

Our study made a preliminary exploration on the relationship between CHD and negative psychological effects, but there are still some shortcomings in our study: first, this study is a retrospective case study, which needs to be confirmed by a larger sample of randomized controlled trials; second, the number of patients included in this study is small and the follow-up time is not long. Therefore, the conclusions of this study need to be confirmed in randomized controlled trials with a larger number of patients in the future.

In conclusion, depression is a meaningful and independent predictor of poor prognosis in CHD patients with stent implantation and the control of risk factors such as depression is very important to improve the prognosis. Therefore, in clinical work, it is suggested to strengthen the screening of depressive disorders in patients with CHD, in addition to routine treatment and nursing during hospitalization, medical staff should timely apply simple and effective assessment tools to find and take active measures to improve the depression of patients.

## Figures and Tables

**Table 1:** Univariate analysis of the incidence of MACE in patients with CHD after stent implantation [*n*%].

Group	MACE (*n* = 32)	No MACE (*n* = 271)	*t*/*χ*^2^	*P*
Age	63.29 ± 13.76	62.28 ± 10.33	*0.380*	*0.705*
Smoking	18 (56.25)	108 (39.85)	*3.168*	*0.076*
Gender (male/female)	27/5	208/63	*0.955*	*0.328*
BMI (kg/m^2^)			*1.279*	*0.258*
<24	12 (37.50)	126 (46.49)		
≥24	20 (62.50)	45 (16.61)		
History of hypertension	23 (71.88)	106 (39.11)	*12.564*	*P* < 0.01
Diabetes history	6 (18.75)	73 (26.94)	*0.995*	*0.318*
History of dyslipidemia	11 (34.38)	84 (31.00)	*0.152*	*0.697*
Family history of premature CHD	2 (6.25)	48 (17.71)	*2.729*	*0.099*
Diagnosis			4.049	*0.256*
STEMI	15 (46.88)	142 (52.40)		
Non-STEMI	4 (12.50)	56 (20.66)		
Unstable angina pectoris	10 (31.25)	63 (23.25)		
Stable angina	3 (9.38)	10 (3.69)		
Number of diseased vessels	2.18 ± 0.83	1.97 ± 0.84	*1.339*	*0.182*
Degree of vascular stenosis (%)	90.45 ± 13.61	91.53 ± 10.48	*0.533*	*0.595*
LVEF (%)	55.46 ± 9.22	56.87 ± 11.49	*0.669*	*0.504*
hsCRP (mg/L)	6.43 ± 6.87	4.83 ± 6.74	*1.267*	*0.206*
Anxiety (0~20)			*8.456*	*P* < 0.01
*Y*	18 (56.25)	83 (30.63)		
*N*	14 (43.75)	188 (69.37)		
Depression (0~20)			*22.763*	*P* < 0.01
*Y*	20 (62.50)	62 (22.88)		
*N*	12 (37.50)	209 (77.12)		
Anxiety combined with depression			*18.449*	*P* < 0.01
*Y*	15 (46.88)	42 (15.50)		
*N*	17 (53.13)	229 (84.50)		

**Table 2:** Cox proportional risk regression analysis variable assignment.

Item	Variable	Assignment	
Dependent variable	MACE	*N* = 0	*Y* = 1
Independent variable	Gender	Male = 1	Female = 2
	BMI	Normal or thin	Overweight or obese
	Smoking	No	Yes
	Hypertension	No	Yes
	Dyslipidemia	No	Yes
	Family history of premature CHD	No	Yes
	Diagnosis	Stable angina = 1	Unstable angina pectoris = 2
		Non-STEM = 3	STEMI = 4
	Anxiety	No	Yes
	Depression	No	Yes
	Anxiety combined with depression	No	Yes

**Table 3:** Cox regression analysis of the effect of anxiety on MACE.

	Uncorrected			Corrected		
	HR	95% CI	*P*	HR	95% CI	*P*
Anxiety	3.181	1.603~6.301	0.001	3.742	1.518~9.173	0.003
Age				1.016	0.971~1.064	0.432
Sex				0.183	0.044~0.833	0.026
BMI				1.535	0.597~3.962	0.373
Smoking				2.281	0.351~2.541	0.912
Hypertension				2.288	0.864~6.067	0.093
Diabetes				0.764	0.279~2.106	0.605
Dyslipidemia				1.481	0.563~3.687	0.447
Family history of premature CHD				0.122	0.107~1.315	0.126
Angina				1.354	0.873~2.124	0.173
Number of diseased vessels				1.366	0.832~2.231	0.215
Degree of diseased vessels				0.971	0.946~41.018	0.341
LVEF (%)				0.976	0.943~1.011	0.163
hsCRP (mg/L)				1.053	1.016~1.106	0.011

**Table 4:** Cox regression analysis of the effect of anxiety combined with depression on MACE.

	Uncorrected			Corrected		
	HR	95% CI	*P*	HR	95% CI	*P*
Anxiety combined with depression	4.642	2.363~9.104	<0.001	3.702	1.576~8.673	0.004
Age				1.024	0.974~1.071	0.421
Sex				0.224	0.051~1.015	0.053
BMI				1.544	0.577~3.701	0.426
Smoking				0.986	0.373~2.574	0.977
Hypertension				2.166	0.823~5.694	0.113
Diabetes				0.763	0.283~2.041	0.592
Dyslipidemia				1.331	0.534~3.291	0.534
Family history of premature CHD				0.454	0.124 ~ 1.643	0.227
Diagnosis				0.743	0.466~1.201	0.224
Number of diseased vessels				1.276	0.783~2.066	0.325
Degree of diseased vessels				0.977	0.943~1.012	0.246
LVEF (%)				0.981	0.953~1.016	0.323
hsCRP (mg/L)				1.036	0.994~1.083	0.075

**Table 5:** COX regression analysis of the effect of anxiety combined with depression on MACE.

Group	HR	95% CI	*P*
A–D − (no anxiety, no depression)	1.001	/	/
A + D − (anxiety, no depression)	2.793	0.914~8.526	0.075
A–D + (no anxiety, depression)	5.734	1.873~17.546	0.003
A + D + (anxiety, depression)	7.303	3.091~17.231	<0.001

## Data Availability

No data were used to support this study.
